The article "Expanding Horizons: A Case Report of Cleft Expansion in the Mixed Dentition Stage" was published in 2023. Journal: Cureus.

# Expanding Horizons: A Case Report of Cleft Expansion in the Mixed Dentition Stage

**DOI:** 10.7759/cureus.51091

**Published:** 2023-12-25

**Authors:** Lovely Bharti, Pallavi Daigavane, Sunita Shrivastav, Ranjit Kamble, Shourya Bharadwaj, Unnati Shirbhate, Aksha Bhargava

**Affiliations:** 1 Orthodontics & Dentofacial Orthopedics, Sharad Pawar Dental College, Datta Meghe Institute of Higher Education and Research, Wardha, IND; 2 Orthodontics and Dentofacial Orthopaedics, Jaipur Dental College and Hospital, Jaipur, IND; 3 Periodontics, Sharad Pawar Dental College, Datta Meghe Institute of Higher Education and Research, Wardha, IND; 4 Oral and Maxillofacial Surgery, Mahatma Gandhi Medical College and Research Institute, Jaipur, IND

**Keywords:** class iii, trihelix expander, palatal fistula, maxillary expansion, cleft lip & palate

## Abstract

A nine-year-old boy with a cleft lip and palate had midface retrusion as a result of maxillary complex growth inhibition. He sought treatment for total crossbite with a Class III skeletal pattern. The maxillary expansion widened the maxilla to improve the sagittal and transverse skeletal relationship. In skeletal Class III patients with a repaired cleft lip and palate, maxillary expansion and protraction usually provide effective improvement. The individual growth of the maxilla and mandible is crucial to the success of the orthopedic procedure.

## Introduction

Cleft palate, a congenital condition marked by a fissure in the roof of the mouth, poses a multifaceted challenge in dental care, particularly during the mixed dentition phase [1]. The amalgamation of orthodontic and surgical interventions becomes paramount for addressing aesthetic concerns and ensuring functional harmony. This case report delves into a pioneering approach to cleft palate management, specifically focusing on palatal expansion in a mixed dentition patient [1,2]. Mixed dentition, characterized by the coexistence of primary and permanent teeth, introduces a dynamic element to treatment planning. The complexities inherent in this phase necessitate innovative strategies to optimize outcomes. Palatal expansion emerges as a pivotal component, offering a transformative pathway to enhance form and function [2]. As we navigate through this case study, the intricacies of the patient's unique presentation, the rationale behind the chosen intervention, and the ensuing success of the palatal expansion will unfold [2,3].

The journey from diagnosis to treatment completion is a testament to the collaborative efforts of orthodontic and surgical disciplines, pushing the boundaries of traditional approaches. This report aims to contribute to the evolving landscape of cleft palate management, shedding light on the efficacy of palatal expansion as a cornerstone in achieving comprehensive and lasting results for mixed dentition patients with cleft palate anomalies [3].

## Case presentation

A nine-year-old boy presented with the chief complaint of a unilateral cleft lip and palate and his major concern was esthetic appearance, malaligned teeth, and speech problems. The patient had a history of lip repair and the closure of palatal fistula at the age of one and four years, respectively. There was no significant medical history. He had a concave facial profile with a flattened nasal tip, shortened columella, an undergrown maxilla, and diminished malar prominence when observed during the extra oral examination (Figure 1).

**Figure 1:** Pre-treatment extraoral photographs: (A) frontal, (B) smiling,(C) profile, (D) worm's view, and (E) bird's eye view

Intra-oral examination revealed a prominent oronasal fistula perforation within palatal scar tissue on the left side, an anterior crossbite with a 2 mm reverse overjet, an open bite (unilateral) on the left side, and all primary teeth except 62,72,73 were present. The arch form of the mandible is in a relatively good condition as compared to the maxillary arch (Figure 2).

**Figure 2:** Pre-treatment intra-oral photograph: (A) frontal view, (B) right lateral view, (C) left lateral view, (D) maxillary occlusal view, and (E) mandibular occlusal view

On radiographic examination, OPG (orthopantomogram) showed developing tooth buds of 11, 12, 13, 23, 24, 32, 33, 34, 35, 37, 43, 44, 45, 47, and supernumerary teeth in the upper left quadrant (Figure 3B); the maxillary occlusal radiograph (Figure 3C) shows 'V' shape arch form with a cleft on the left side. The cephalometric analysis concluded the presence of a skeletal Class III pattern with a maxilla, vertical growth pattern, clockwise rotation of maxilla and mandible, retroclined upper incisors, normally inclined lower incisors, and the Class III soft-tissue profile was revealed by cephalometric analysis (Figure 3A).

**Figure 3:** Pre-treatment radiographs: (A) lateral cephalogram, (B) OPG (orthopantomogram), and (C) maxillary occlusal

Based on the above observations, the patient had a vertical growth pattern with a class III skeletal profile. In the current case, the hypoplastic growth of the maxilla made it appear retrognathic, while the mandible was normal. Initially, intercanine and intermolar widths were 22mm and 40mm respectively. The treatment modality, in this case, included anterior and posterior maxillary expansions followed by extraction of supernumerary teeth, alveolar bone grafting, arch leveling, and alignment. Fabrication of a trihelix expander was done which was the initial step in the treatment. The expander was cemented within the maxillary arch (Figure 4) with the help of glass ionomer cement, and after every four weeks, it was activated (both posterior coils were opened to a quarter of their diameter) using a three-prong plier to obtain an expansion of the maxillary arch. After six months of activation, maxillary anterior and posterior expansion was achieved (Figure 6). After expansion, a positive overjet can be appreciated (Figure 5B, Figure 6B). After six months, both anterior and posterior expansion took place, and there was an increase in intercanine width (Figure 6D). Comparable expansion can be recognized clinically (Figure 7) and radiographically where both intercanine (27mm) and intermolar widths (48mm) have been increased (Figure 8). However, the lateral cephalogram and orthopantomogram show no significant changes post expansion (Figure 9) as the changes were mainly in the transverse plane. 

**Figure 4:** After placement of tri-helix expander (A) maxillary arch, (B) frontal view, (C) right lateral view, and (D) left lateral view

**Figure 5:** Post-expansion extraoral photographs: (A) frontal, (B) smiling, (C) profile, (D) worm's view, and (E) bird's eye view

**Figure 6:** Post-expansion intra-oral photographs: (A) frontal view, (B) right lateral view, (C) left lateral view, (D) maxillary occlusal view, and (E) mandibular occlusal view

**Figure 7:** Sequential photographs of maxillary arch: (A) before expansion, (B) during expansion with trihelix expander, and (C) post-expansion

**Figure 8:** Comparison of maxillary occlusal radiograph (A) pre-treatment and (B) post-expansion

**Figure 9:** Post-expansion radiographs: (A) lateral cephalogram, (B) orthopantomogram (OPG), and (C) maxillary occlusal

## Discussion

The complex nature of cleft palate management in mixed dentition patients demands a comprehensive understanding of the complex relationships between skeletal, dental, and soft tissue structures [3]. In this case, palatal expansion emerges as a pivotal strategy, demonstrating its multifaceted efficacy in addressing both functional and aesthetic dimensions. [4].

From a functional standpoint, the application of palatal expansion was strategically employed to navigate the challenges posed by the mixed dentition phase [5]. By creating additional space for the eruption of permanent dentition, the intervention reduced crowding and malocclusion issues and played a crucial role in optimizing occlusal relationships and overall dental alignment. This functional success is pivotal, as it resolves immediate concerns and sets the stage for subsequent orthodontic adjustments and long-term stability [6].

Rapid palatal expansion generates greater sutural forces in a short period of time. These strong forces maximize the skeletal expansion of the midpalatal suture prior to any dental movement or physiological sutural adjustment. When RME is performed in the prepubertal period or during puberty, skeletal and dental effects are easily achieved, and relapse is rare. Slow expansion of the constricted palate is possible in cleft palate cases because the buttressing effect of the zygoma is absent [7].

Trihelix demonstrated the effectiveness of using a trihelix appliance with push coils to reciprocally move molars and incisors apart to create enough space. The trihelix is a modified quadhelix fixed expander made of 0.028 stainless steel wire with three helices instead of four, making it less bulky than the quadhelix and suitable for cases of severe palatal constriction where another palatal expander cannot be fitted. Because there was no room in the palatal space for a quadhelix due to the presence of severely palatally displaced teeth, the present case is the best example of such an indication for the use of a trihelix expander [8].

Aesthetic considerations are equally paramount, especially in the context of cleft palate patients undergoing treatment during the mixed dentition phase. The correction of posterior crossbites and enhancements in arch form resulting from palatal expansion contributes significantly to achieving a more symmetrical and harmonious smile. Also expanding the arch in the mixed dentition phase helps the surgeon to know the actual defect size of a cleft in the palate, minimizing the formation of a fistula later [8]. The transformative impact on facial aesthetics is not merely a cosmetic enhancement but holds profound implications for the patient's psychosocial well-being [9].

In this case, the success of palatal expansion is also a testament to the power of interdisciplinary collaboration between orthodontic and surgical specialties [9]. The seamless integration of expertise and coordinated efforts in treatment planning and execution allowed for a dynamic approach, accommodating the unique challenges presented by mixed dentition cleft palate cases. Regular communication between the specialists facilitated timely adjustments to the treatment plan, emphasizing the importance of a holistic and adaptive approach to achieving optimal outcomes [10]. In considering the longevity of treatment success, the case underscores the importance of ongoing follow-up assessments. Monitoring dental and skeletal changes over time is crucial to ensuring the stability of the intervention and validating the lasting impact of palatal expansion in mixed dentition cleft palate patients [11].

As the field of cleft palate management continues to evolve, this case contributes to the broader narrative, emphasizing the immediate success of palatal expansion and the adaptability of treatment approaches to the unique needs of mixed dentition patients. This case highlights the transformative potential of innovative strategies in optimizing both functional and aesthetic outcomes, thereby shaping the future landscape of comprehensive cleft palate care [12].

## Conclusions

The successful use of palatal expansion in this mixed dentition cleft palate case demonstrated its functional and aesthetically transformative impact. The intervention addressed immediate concerns, laid the groundwork for future orthodontic adjustments, and significantly improved the patient's smile and facial aesthetics. In navigating the complexities of mixed dentition cases, the collaborative interdisciplinary approach between orthodontic and surgical specialties proved invaluable. This case illustrates the changing landscape of cleft palate care, emphasizing innovative strategies, adaptability, and transformative potential for improved patient outcomes.
